The article "Long non-coding RNA SNHG1 protects human AC16 cardiomyocytes from doxorubicin toxicity by regulating miR-195/Bcl-2 axis" was retracted in 2023. Reasons: duplicated images; signs of a paper mill; concerns about the images.

# Long non-coding RNA SNHG1 protects human AC16 cardiomyocytes from doxorubicin toxicity by regulating miR-195/Bcl-2 axis

**DOI:** 10.1042/BSR20191050

**Published:** 2019-07-26

**Authors:** Sisi Chen, Jichun Wang, Yanli Zhou

**Affiliations:** 1 Department of Cardiology, Renmin Hospital of Wuhan University, Wuhan 430060, China; 2 Cardiovascular Research Institute, Wuhan University, Wuhan 430060, China; 3 Hubei Key Laboratory of Cardiology, Wuhan 430060, China

**Keywords:** apoptosis, cardiotoxicity, doxorubicin, long non-coding RNA SNHG1, miR-195

## Abstract

Doxorubicin (DOX) is a highly effective anti-tumor drug, but its cardiotoxicity largely restricts its clinical application. The present study was designed to explore whether *in vitro* DOX toxicity in AC16 cardiomyocytes can be regulated by long non-coding RNA (lncRNA) small nucleolar RNA host gene 1 (SNHG1) and to elucidate the underlying mechanisms. We found that DOX treatment led to severe damage in AC16 cells through decreasing cell viability and increasing cell apoptosis. DOX treatment also reduced the expression of SNHG1 in AC16 cells, and overexpression of SNHG1 alleviated the increased apoptosis in DOX-treated AC16 cells. Moreover, we found that SNHG1 could counteract the inhibitory effect of miR-195 on Bcl-2, and miR-195 restoration blocked the beneficial effect of SNHG1 against DOX toxicity in AC16 cells. In short, the present study provided convincing evidence that SNHG1 protects human AC16 cardiomyocytes from DOX toxicity partly by regulating miR-195/Bcl-2 axis.

## Introduction

Cancer is the main cause of deaths worldwide. Doxorubicin (DOX), an anthracycline antibiotic derived from *Streptomyces*, is one of the most powerful and widely used anti-tumor drugs [1]. However, the clinical application of this drug is largely limited by the toxic side effects on healthy human organs, specifically heart [2]. Approximately 10% of patients treated with DOX or its derivatives will develop cardiac complications [3]. Accordingly, there is a growing need to develop effective therapies against DOX cardiotoxicity.

Long non-coding RNAs (lncRNAs), a group of RNA molecules greater than 200 nucleotides in length with limited protein-coding potential, have been recently identified as a critical player in many human diseases, including cardiovascular disorders [4]. LncRNA small nucleolar RNA host gene 1 (SNHG1), located in human chromosome 11, was found to be aberrantly expressed in a wide variety of human cancers [5]. In addition, Zhang et al. [6] reported that SNHG1 attenuated the effects of H_2_O_2_ on the viability and apoptosis of human cardiomyocytes. In this study, using *in vitro* DOX-treated AC16 cardiomyocytes, our major purpose was to explore whether DOX toxicity can be regulated by SNHG1 and to elucidate the underlying mechanisms.

The article "Long non-coding RNA SNHG1 protects human AC16 cardiomyocytes from doxorubicin toxicity by regulating miR-195/Bcl-2 axis" was retracted in 2023. Reasons: duplicated images; signs of a paper mill; concerns about the images.

## Materials and methods

### Cell culture and treatments

The human cardiomyocyte-like AC16 cells [7], obtained from American Type Culture Collection (ATCC; Rockville, MD, U.S.A.), were cultured in Dulbecco’s Modified Eagle’s Medium (DMEM; Invitrogen, Carlsbad, CA, U.S.A.) containing 10% FBS (Biowest, Loire, France) and 100 mg/ml penicillin/streptomycin in a humidified atmosphere of 5% CO_2_ at 37°C.

DOX (Sangon Biotech Co., Ltd., Shanghai, China) was dissolved in DMSO and diluted with cell culture medium to achieve a final concentration of 5 μM.

For SNHG1 overexpression, the full-length cDNA of SNHG1 was synthesized and cloned into the expression vector pcDNA3.1 (Invitrogen). An empty vector served as a negative control (NC). The short interfering RNA targeting SNHG1 (si-SNHG1) and NC (si-NC) were chemically synthesized by GenePharma Co., Ltd. (Shanghai, China), and their sequences were listed as follows: si-SNHG1, 5′-GAAACAGCAGUUGAGGGUUUGCUGU-3′; si-NC, 5′-GAUCAUACGUGCGAUCAGA-3′. The specific mimics, inhibitor and the corresponding NC for miR-195 were chemically synthesized by RiboBio Co., Ltd. (Guangzhou, China). Two hours before DOX stimulation, cells were seeded in six-well plates and the transfection was performed by using Lipofectamine 2000 reagent (Invitrogen).

### Cell counting kit-8 assay

Cell viability was determined by Cell Counting Kit-8 (CCK-8; Dojindo Laboratories, Kumamoto, Japan). Briefly, after treatments, CCK-8 solution (10 μl) was added to each well, and the plates were incubated for additional 1 h. The absorbance of each well was measured at 450 nm using a microplate reader (MultiskanEX, Lab systems, Helsinki, Finland).

### Cell apoptosis analysis

Cell apoptosis was determined by Annexin V-FITC Apoptosis Detection Kit (BD Biosciences, San Jose, CA, U.S.A.). Briefly, after treatments, cells were washed in PBS and re-suspended in 100 μl binding buffer. Then, cells were stained with 5 μl Annexin V-FITC and 1 μl PI. Followed by incubation for 1 h in the dark, cells were then subjected to FACScan flow cytometer (BD Biosciences) equipped with CellQuest software.

### RT-qPCR analysis

Total RNA samples were extracted using TRIzol reagent (Invitrogen). One of total RNA was then reverse-transcribed into cDNA by using the PrimeScript RT reagent Kit (TaKaRa, Dalian, China), and qPCR analysis was performed using the SYBR Premix ExTaq II kit (TaKaRa) on a 7500HT Real-Time PCR System (Applied Biosystems, Foster City, CA, U.S.A.). The relative gene expression was calculated using the 2^−ΔΔ*C*^_t_ method [8], and GAPDH or U6 was used as an internal control. The sequences of primers were shown as follows: SNHG1, forward primer: 5′-ACGTTGGAACCGAAGAGAGC-3′ and reverse primer: 5′-GCAGCTGAATTCCCCAGGAT-3′; GAPDH, forward primer: 5′-CTCTGCTCCTCCTGTTCGAC-3′ and reverse primer: 5′-CGACCAAATCCGTTGACTCC-3′; miR-195, RT: 5′-GTCGTATCCAGTGCAGGGTCCGAGGTATTCGCACTGGATACGACGCCAAT-3′, forward primer: 5′-GGCTAGCAGCACAGAAAT-3′ and reverse primer: 5′-GTGCAGGGTCCGAGGT-3′; U6, RT: 5′-GTCGTATCCAGTGCAGGGTCCGAGGTATTCGCACTGGATACGACAAAATA-3′, forward primer: 5′-CTCGCTTCGGCAGCACATATACT-3′ and reverse primer: 5′-ACGCTTCACGAATTTGCGTGTC-3′.

The article "Long non-coding RNA SNHG1 protects human AC16 cardiomyocytes from doxorubicin toxicity by regulating miR-195/Bcl-2 axis" was retracted in 2023. Reasons: duplicated images; signs of a paper mill; concerns about the images.

### Western blot analysis

Total protein was extracted using radioimmunoprecipitation-assay buffer (Beyotime, Shanghai, China). Equal amounts of protein samples were separated by SDS/PAGE and then electrophoretically transferred to PVDF membranes (Millipore, Billerica, MA, U.S.A.). The membranes were probed with the specific primary antibodies against Bcl-2 (dilution, 1:1000; Abcam, Cambridge, MA, U.S.A.), Bax (dilution, 1:1000; Abcam), cleaved caspase-3/caspase-3 (dilution, 1:1000; Cell Signaling Technology, Danvers, MA, U.S.A.) and GAPDH (dilution, 1:2000; Santa Cruz Biotechnology, Dallas, TX, U.S.A.) at 4°C overnight, followed by incubation with HRP-conjugated secondary antibody (dilution, 1:10000; Santa Cruz Biotechnology). Immunoreactive bands were visualized using the enhanced chemiluminescence reagents (Bio-Rad, Hercules, CA, U.S.A.), and GAPDH was considered as an inner loading control.

### Dual-luciferase reporter assay

The fragment of SNHG1 or Bcl-2 carrying a putative miR-195-binding site was amplified by PCR and inserted into the psiCHECK-2 luciferase reporter vector (Promega, Madison, WI, U.S.A.). The binding sites were mutated using a Mut Express II Fast Mutagenesis kit (Vazyme, Piscataway, NJ, U.S.A.). Cells were seeded in 24-well plates and co-transfected with the luciferase reporter plasmid and miR-195 mimics or NC using Lipofectamine 2000. After 48 h, the cells were lysed, and the luciferase activities were measured using the dual-luciferase reporter assay system (Promega).

### Statistical analysis

All statistical analyses were performed using GraphPad Prism (version 6.01) software (GraphPad Software, Inc., La Jolla, CA, U.S.A.). Data were expressed as mean ± standard deviation (SD) of three repeated experiments, each consisting of three culture plates (*n*=9). The difference between groups was determined by Student’s *t* test or one-way ANOVA. All *P*-values were two sided, and *P*<0.05 was statistically significant.

## Results

### DOX reduces SNHG1 expression in AC16 cells

First, as shown in Figure 1A, the exposure of AC16 cells to DOX for 24 h induced remarkable cytotoxicity, leading to a decrease in cell viability. In addition, the apoptosis rate of AC16 cells was strikingly increased after DOX treatment (Figure 1B). Western blot analysis also showed that the expression of pro-apoptotic proteins (Bax and cleaved caspase-3) was increased, whereas the expression of anti-apoptotic protein (Bcl-2) was decreased in DOX-treated AC16 cells (Figure 1C). Moreover, as indicated by RT-qPCR analysis, DOX treatment remarkably decreased SNHG1 expression in AC16 cells (Figure 1D).

The article "Long non-coding RNA SNHG1 protects human AC16 cardiomyocytes from doxorubicin toxicity by regulating miR-195/Bcl-2 axis" was retracted in 2023. Reasons: duplicated images; signs of a paper mill; concerns about the images.

**Figure 1:** DOX reduces SNHG1 expression in AC16 cells (**A**) Effect of DOX treatment on AC16 cell viability, detected by CCK-8 assay. (**B**) Effect of DOX treatment on AC16 cell apoptosis, detected by flow cytometric analysis. (**C**) Effect of DOX treatment on apoptosis-related protein expression in AC16 cells, detected by Western blot analysis. (**D**) Effect of DOX treatment on SNHG1 expression in AC16 cells, detected by RT-qPCR analysis. Each experiment was repeated three times. *P<0.05 vs. control cells.

### SNHG1 alleviates DOX toxicity in AC16 cells

To further investigate the role of SNHG1 in DOX toxicity, SNHG1 was then overexpressed in DOX-treated AC16 cells, and the successful transfection was verified by RT-qPCR analysis (Figure 2A). As shown in Figure 2B, SNHG1 overexpression significantly alleviated DOX toxicity by increasing the AC16 cell viability. Moreover, SNHG1 overexpression also markedly reduced the apoptosis rate of DOX-treated AC16 cells (Figure 2C). As revealed by Western blot analysis, SNHG1 overexpression increased the Bcl-2/Bax expression ratio and suppressed the cleavage of caspase-3 in DOX-treated AC16 cells (Figure 2D).

**Figure 2:** SNHG1 alleviates DOX toxicity in AC16 cells (**A**) Transfection efficacy was verified by RT-qPCR analysis. (**B**) Effect of SNHG1 overexpression on the viability of DOX-treated AC16 cells. (**C**) Effect of SNHG1 overexpression on the apoptosis of DOX-treated AC16 cells. (**D**) Effect of SNHG1 overexpression on the expression levels of apoptosis-related proteins in DOX-treated AC16 cells. Each experiment was repeated three times. *P<0.05 vs. empty vector-transfected cells.

### SNHG1 acts as a competing endogenous RNA for miR-195 in AC16 cells

By using the Starbase database (http://starbase.sysu.edu.cn/index.php), miR-195 was predicted to directly bind to SNHG1, with the binding sequences shown in Figure 3A. To verify the prediction, dual-luciferase reporter assay was then performed, and the results demonstrated that miR-195 mimics decreased the luciferase activity of SNHG1-WT but had no obvious effect on SNHG1-MUT in AC16 cells (Figure 3B). We also found that SNHG1 overexpression decreased, whereas SNHG1 knockdown increased miR-195 expression in AC16 cells (Figure 3C).

The article "Long non-coding RNA SNHG1 protects human AC16 cardiomyocytes from doxorubicin toxicity by regulating miR-195/Bcl-2 axis" was retracted in 2023. Reasons: duplicated images; signs of a paper mill; concerns about the images.

**Figure 3:** SNHG1 acts as a competing endogenous RNA for miR-195 in AC16 cells (**A**) Bioinformatical predication of interaction between SNHG1 and miR-195. (**B**) Relative luciferase activity of AC16 cells co-transfected with SNHG1-WT or SNHG1-MUT and miR-195 mimics or NC. (**C**) Effect of SNHG1 overexpression or knockdown on miR-195 expression in AC16 cells. (**D**) Bioinformatical predication of interaction between miR-195 and Bcl-2. (**E**) Relative luciferase activity of AC16 cells co-transfected with Bcl-2-WT or Bcl-2-MUT and miR-195 mimics or NC. (**F**) Effect of miR-195 overexpression or inhibition on Bcl-2 protein expression in AC16 cells. Each experiment was repeated three times. *P<0.05 vs. NC-transfected cells; ^#^*P*<0.05 vs. empty vector-transfected cells; ^∧^*P*<0.05 vs. si-NC-transfected cells.

Utilizing the TargetScan database (http://www.targetscan.org), Bcl-2 was predicted as a potential target gene of miR-195 (Figure 3D), and this prediction was confirmed by dual-luciferase reporter assay, as the luciferase activity was markedly reduced in AC16 cells by co-transfection with Bcl-2-WT and miR-195 mimics (Figure 3E). Besides, as shown in Figure 3F, miR-195 overexpression decreased, whereas miR-195 inhibition increased Bcl-2 protein expression in AC16 cells.

### miR-195 inhibition alleviates DOX toxicity in AC16 cells

Furthermore, as shown in Figure 4A, miR-195 is significantly up-regulated after DOX treatment in AC16 cells. We then found that the increased apoptosis rate of DOX-treated AC16 cells was also diminished by miR-195 inhibition (Figure 4B), whereas CCK-8 assay indicated that miR-195 inhibition rescued the impaired viability of DOX-treated AC16 cells (Figure 4C).

**Figure 4:** miR-195 inhibition alleviates DOX toxicity in AC16 cells (**A**) Effect of DOX treatment on miR-195 expression in AC16 cells. (**B**) Effect of miR-195 inhibition on the apoptosis of DOX-treated AC16 cells. (**C**) Effect of miR-195 inhibition on the viability of DOX-treated AC16 cells. Each experiment was repeated three times. *P<0.05 vs. control cells; ^#^*P*<0.05 vs. NC-transfected cells.

### miR-195 blocks the beneficial role of SNHG1 in DOX-treated AC16 cells

We subsequently carried out rescue experiments, and the results showed that co-transfection with miR-195 mimics obviously blocked the beneficial role of SNHG1, through increasing the apoptosis (Figure 5A) and decreasing the viability (Figure 5B) of DOX-treated AC16 cells.

**Figure 5:** miR-195 blocks the beneficial role of SNHG1 in DOX-treated AC16 cells (**A**) The apoptosis of DOX-treated AC16 cells after co-transfection. (**B**) The viability of DOX-treated AC16 cells after co-transfection. Each experiment was repeated three times. *P<0.05 vs. SNHG1+NC-transfected cells.

The article "Long non-coding RNA SNHG1 protects human AC16 cardiomyocytes from doxorubicin toxicity by regulating miR-195/Bcl-2 axis" was retracted in 2023. Reasons: duplicated images; signs of a paper mill; concerns about the images.

## Discussion

DOX cardiotoxicity remains a tough problem for both cardiologists and oncologists, and the underlying mechanisms have been extensively studied since DOX was first used. Recently, lncRNAs have attracted increasing attention due to their regulatory role in DOX cardiotoxicity. For example, LINC00339 aggravates DOX-induced cardiomyocyte apoptosis [9], and FOXC2-AS1 was down-regulated in heart tissues of mice with DOX cardiotoxicity [10]. In this study, the effects of SNHG1 on DOX-treated AC16 cardiomyocytes were studied.

The heart is composed of various types of cells, and cardiomyocyte is a classical cellular target of DOX [11]. Apoptosis, a type of programmed cell death, plays an essential role in the pathogenesis of DOX cardiotoxicity [12]. Myocardial apoptosis causes loss of myocytes and impairment of heart function. Hence, identification of effective methods to suppress DOX-induced apoptosis of cardiomyocytes is imperative. In the present study, we also identified a significant increase in the apoptosis rates of AC16 cells after DOX stimulation, which was further diminished by SNHG1 overexpression.

We then explored the possible mechanisms underlying the beneficial role of SNHG1. MicroRNAs (miRNAs), another type of noncoding RNA, are well characterized. A wealth of studies indicate that lncRNAs can serve as competing endogenous RNAs (ceRNAs) to regulate the expression and activity of miRNA [13,14]. miR-195, a critical regulator in cardiac physiology, is overexpressed in STZ-induced diabetic mouse hearts and hypoxia/reoxygenation-treated H9c2 cells [15,16]. In the present study, we provided several lines of evidence to indicate that, in DOX-treated AC16 cells, miR-195 expression was increased, and SNHG1 might act as a ceRNA for miR-195 to enhance the expression of target gene Bcl-2, thereby alleviating the DOX toxicity.

In conclusion, the present study, for the first time, demonstrated that SNHG1 could protect human AC16 cardiomyocytes from DOX toxicity partly by regulating miR-195/Bcl-2 axis. Our findings provided a possible molecular mechanism underlying DOX cardiotoxicity, which will gives a new direction for its treatment.

## Abbreviations

Bcl-2: B-cell lymphoma-2
CCK-8: Cell Counting Kit-8
ceRNA: competing endogenous RNA
DOX: doxorubicin
FOXC2-AS1: FOXC2-antisense RNA 1
GAPDH: Glyceraldehyde-3-phosphate dehydrogenase
HRP: Horse radish peroxidase
lncRNA: long non-coding RNA
miRNA: microRNA
PI: Propidium iodide
qPCR: Quantitative PCR
RT-qPCR: Reverse transcription-quantitative PCR
SNHG1: small nucleolar RNA host gene 1
